The article "Multidisciplinary Approaches to Limb Salvage in Traumatic Extremity Injuries From Emergency Triage to Definitive Vascular, Orthopedic, and Reconstructive Surgery: A Systematic Review" was retracted in 2025. Reasons: unreliable results or conclusions; concerns about the authorship.

# Multidisciplinary Approaches to Limb Salvage in Traumatic Extremity Injuries From Emergency Triage to Definitive Vascular, Orthopedic, and Reconstructive Surgery: A Systematic Review

**DOI:** 10.7759/cureus.86252

**Published:** 2025-06-17

**Authors:** Nabila Issa Youssouf, Huba Ali Khan, Asma Ahmed Osman Mohamed, Mohamed Bahaa Aboelsebaa Othman, Mahmoud Hassan Fadul Ismail, Ahmed A Hassan, Aliaa H Alkhazendar, Jarallah H. J. Alkhazendar, Monezahe Zehra, Deewan Aakash

**Affiliations:** 1 Surgery, International University of Africa, Khartoum, SDN; 2 Emergency Medicine, Ziauddin University, Karachi, PAK; 3 Surgery, Burjeel Medical City, Abu Dhabi, SAU; 4 Vascular Surgery, Nasser Institute Hospital for Research and Treatment, Cairo, EGY; 5 International Public Health, Royal Infirmary of Edinburgh, Edinburgh, GBR; 6 Orthopedics and Trauma, Suez Canal University Hospital, Ismailia, EGY; 7 Surgery, Islamic University of Gaza, Gaza, PSE; 8 General and Emergency Surgery, East and North Hertfordshire NHS Trust, Lister Hospital, Stevenage, GBR; 9 Surgery, Abbasi Shaheed Hospital, Karachi, PAK; 10 Surgery, Liaquat National Hospital, Karachi, PAK

**Keywords:** amputation, complex extremity trauma, limb reconstruction, limb salvage, mangled limb, multidisciplinary team, orthoplastic surgery, trauma management, trauma surgery outcomes, vascular surgery

## Abstract

This systematic review explores the impact of multidisciplinary team (MDT) approaches in the management of complex limb injuries, comparing limb salvage and amputation outcomes across diverse trauma settings. Drawing from six recent studies involving both acute and chronic extremity trauma, the findings highlight consistent benefits of coordinated care involving orthopedic, vascular, and plastic surgery specialties. These include reduced flap loss, faster time to definitive fixation, improved functional recovery, and enhanced decision-making regarding salvage versus amputation. While functional and psychological outcomes following salvage and amputation were often comparable, early MDT involvement improved wound healing and lowered short-term mortality rates in select patient groups. Variability in outcomes was influenced by institutional resources, timing of intervention, and patient comorbidities. Scoring systems such as the Mangled Extremity Severity Score (MESS) and the Mangled Extremity Syndrome Index (MESI) aided but did not replace clinical judgment. Overall, the integration of multidisciplinary pathways into trauma care enhances outcome quality and supports patient-centered decision-making in complex limb trauma cases.

## Introduction and background

Traumatic extremity injuries are a significant global health concern, especially among young and active individuals. These injuries often result from high-energy incidents such as road traffic accidents (RTAs), falls from height, industrial trauma, or military combat [1]. They commonly involve multiple tissue types, including bone fractures, vascular disruption, nerve injury, and extensive soft tissue damage. Managing such complex injuries requires not only immediate lifesaving and limb-saving interventions but also long-term planning for rehabilitation and function preservation [2]. Over the years, the approach to limb salvage has shifted from isolated surgical decisions to a more collaborative, team-based strategy. Multidisciplinary involvement, bringing together orthopedic, vascular, and plastic surgeons with trauma specialists and rehabilitation teams, has shown promising results [3]. Early debridement, timely revascularization, stable fracture fixation, and strategic soft tissue coverage all play vital roles. Coordinated care helps reduce complication rates such as infection, flap loss, and delayed healing. Despite advancements, the literature remains variable, with many studies differing in methodology, definitions of limb salvage, and outcome measurement.

The article "Multidisciplinary Approaches to Limb Salvage in Traumatic Extremity Injuries From Emergency Triage to Definitive Vascular, Orthopedic, and Reconstructive Surgery: A Systematic Review" was retracted in 2025. Reasons: unreliable results or conclusions; concerns about the authorship.

This systematic review aims to evaluate the role and clinical outcomes of multidisciplinary approaches to limb salvage in traumatic extremity injuries. It assesses whether coordinated care involving multiple specialties leads to better patient outcomes when compared to conventional or single-specialty management, including primary amputation. The review explores the full spectrum of care from emergency triage to definitive orthopedic, vascular, and reconstructive procedures. Outcomes of interest include limb salvage rates, time to fixation, infection and complication rates, functional recovery, and overall patient quality of life.

## Review

Materials and methods

Study Design

This systematic review was designed to evaluate the clinical effectiveness and patient-centered outcomes of multidisciplinary approaches in the management of traumatic limb injuries. The review followed the Preferred Reporting Items for Systematic Reviews and Meta-Analyses (PRISMA) guidelines [4] to ensure methodological rigor, transparency, and replicability.

Eligibility Criteria

The inclusion criteria were developed using the PICO framework [5]. The Population (P) included adult patients with traumatic or ischemic limb injuries, both acute (e.g., Gustilo IIIb fractures and military trauma) and chronic (e.g., diabetic foot and limb-threatening ischemia). Interventions (I) required the involvement of multidisciplinary teams (MDTs), defined as the coordinated participation of at least two specialties such as orthopedic surgery, vascular surgery, plastic/reconstructive surgery, or rehabilitation. Comparisons (C), where applicable, included single-specialty or conventional care. The Outcomes (O) of interest were amputation rates, flap success, time to debridement or fixation, one-year mortality, wound healing, functional status, and patient-reported psychological outcomes. Only peer-reviewed, English language studies with full-text access were considered. Case reports, conference abstracts, editorials, and non-clinical articles were excluded.

The article "Multidisciplinary Approaches to Limb Salvage in Traumatic Extremity Injuries From Emergency Triage to Definitive Vascular, Orthopedic, and Reconstructive Surgery: A Systematic Review" was retracted in 2025. Reasons: unreliable results or conclusions; concerns about the authorship.

Search Strategy

A structured electronic search was conducted across PubMed, MEDLINE, and Google Scholar for articles published between January 2015 and April 2025. Search terms included combinations of “multidisciplinary limb salvage,” “orthoplastic surgery,” “amputation versus reconstruction,” “complex limb trauma,” “vascular injury,” “flap coverage,” and “limb-threatening extremity injuries.” The reference lists of relevant articles were hand-screened to identify additional eligible studies.

Study Selection

After deduplication, two reviewers independently screened titles and abstracts to identify relevant studies. The full texts of potentially eligible articles were reviewed in detail. Disagreements during the selection process were resolved through discussion and mutual consensus. A total of six studies were included in the final review after applying all inclusion and exclusion criteria.

Data Extraction

Key data were extracted independently by two authors using a standardized data extraction form. The following variables were collected: first author and year, study design, patient population and demographics, type of limb trauma, nature of the multidisciplinary intervention, comparison group (if any), specialties involved, outcomes assessed (e.g., time to debridement, flap loss, functional recovery, amputation rate, and mortality), and major conclusions.

Quality Assessment

Each study underwent an independent quality assessment based on its design. Narrative reviews were assessed using the Scale for the Assessment of Narrative Review Articles (SANRA) [6], emphasizing clarity, justification of relevance, and comprehensiveness. Observational and retrospective cohort studies were evaluated using the NIH Quality Assessment Tool [7] for Observational Cohort and Cross-Sectional Studies, focusing on study population, exposure and outcome assessment, and statistical adjustment. The systematic review was appraised with the A Measurement Tool to Assess Systematic Reviews 2 (AMSTAR 2) tool [8], and limited elements of Grading of Recommendations, Assessment, Development and Evaluation (GRADE) were applied for the meta-analysis. This multi-tool approach ensured that each study was assessed appropriately based on its methodological design.

The article "Multidisciplinary Approaches to Limb Salvage in Traumatic Extremity Injuries From Emergency Triage to Definitive Vascular, Orthopedic, and Reconstructive Surgery: A Systematic Review" was retracted in 2025. Reasons: unreliable results or conclusions; concerns about the authorship.

Data Synthesis

Given the heterogeneity in study design, interventions, outcome definitions, and populations, a narrative synthesis approach was adopted. The results were categorized thematically under the following domains: clinical decision-making, surgical outcomes, functional and psychological recovery, and timing of interventions. Tabular summaries were used to present study characteristics and comparative findings, with particular emphasis on elements that directly influence clinical decision-making in limb salvage versus amputation.

Results

Study Selection Process

The study selection process is summarized in Figure 1. A total of 302 records were initially identified through structured searches across three databases: PubMed (n = 96), MEDLINE (n = 88), and Google Scholar (n = 118). After removing 68 duplicate records, 234 unique articles remained for title and abstract screening. Of these, 152 articles were excluded based on irrelevance to the topic or lack of clinical applicability, leaving 82 full-text reports for retrieval. However, 17 could not be accessed, and the remaining 65 articles underwent full-text review. Following the application of the inclusion and exclusion criteria, 59 studies were excluded due to reasons such as being case reports, conference abstracts, editorials, and non-clinical studies, language or access barriers, or lacking a multidisciplinary approach. Ultimately, six studies met the criteria and were included in the final systematic review.

**Figure 1:** PRISMA flow diagram outlining the study selection process for the systematic review PRISMA: Preferred Reporting Items for Systematic Reviews and Meta-Analyses

Characteristics of the Selected Studies

As shown in Table 1, the included studies varied in design, populations, trauma types, and outcome measures but consistently examined the impact of multidisciplinary approaches in limb salvage. Most studies focused on acute or chronic limb-threatening injuries, including diabetic foot complications, crush injuries, vascular trauma, and polytrauma scenarios. Interventions generally involved coordinated care by multiple surgical and medical specialties, such as orthopedic, vascular, plastic, and emergency medicine, with some incorporating psychological and perioperative support. Despite heterogeneity in settings and specific interventions, all studies reported clinical benefits of multidisciplinary care, including improved flap success rates, reduced time to surgical milestones, better functional outcomes, and lower complication or mortality rates. This reinforces the growing consensus that multidisciplinary teamwork enhances decision-making and overall patient recovery in complex extremity trauma.

The article "Multidisciplinary Approaches to Limb Salvage in Traumatic Extremity Injuries From Emergency Triage to Definitive Vascular, Orthopedic, and Reconstructive Surgery: A Systematic Review" was retracted in 2025. Reasons: unreliable results or conclusions; concerns about the authorship.

**Table 1:** Characteristics of the selected studies MDT: multidisciplinary team, FTT: free tissue transfer, LOS: length of stay, RTA: road traffic accident, LE: lower extremity, MLT: multidisciplinary limb team, OR: odds ratio, DCO: damage control orthopedics, CTA: computed tomography angiography, MESS: Mangled Extremity Severity Score, MESI: Mangled Extremity Syndrome Index, NISSSA: Nerve Injury, Ischemia, Soft Tissue Injury, Skeletal Injury, Shock, and Age, TMR: targeted muscle reinnervation

First author (year)	Study design	Population	Type of trauma	Intervention (multidisciplinary approach)	Comparison (if any)	Surgical specialties involved	Outcomes measured	Key findings
Bridgeman and Crist (2022) [9]	Narrative/institutional case overview	Patients with acute and chronic traumatic limb injuries	Acute and chronic traumatic extremity injuries	Integrated team (orthopedic trauma, microsurgeons, vascular, neurosurgery, infectious disease, perioperative medicine, and psychology)	Not directly compared; limb salvage versus amputation discussed	Orthopedic, plastic/reconstructive, vascular, and neurosurgery	Limb salvage feasibility, decision-making quality, and outcomes	MDT improved outcomes, decision-making, and patient recovery. 56% regained sensation; TMR technique reduced amputation pain.
Li et al. (2024) [10]	Retrospective observational study	300 patients, mean age: 55.9, 70.7% male patients	Atraumatic chronic lower limb wounds (mostly diabetic and vascular)	Multidisciplinary preoperative optimization, intraoperative FTT, postoperative wound care, and systemic disease management	No comparison group (single-arm study)	Plastic surgery, vascular medicine, endocrinology, and nephrology	Flap success, amputation rate, and hospital and postoperative LOS	The flap success rate was 96.3%; amputation was 12.7%. Highlights the need for preoperative optimization and MDT follow-up.
Kawaji et al. (2025) [11]	Retrospective cohort study	471 patients undergoing major LE amputations (2014-2021)	Chronic limb-threatening ischemia	MDT limb salvage program implementation	Pre-MLT versus post-MLT groups	Vascular surgery and MDT limb salvage	Revascularization, minor amputation/debridement, and one-year mortality	Pre-amputation revascularization unchanged; one-year mortality post-amputation significantly reduced (OR: 0.54; p = 0.002).
Nayar et al. (2023) [12]	Systematic review (15 studies, 6,113 patients)	6,113 upper limb trauma patients (5,972 salvage and 141 amputation)	Severe upper limb trauma (crush and nerve/vascular injury)	Evaluation of scoring tools and outcomes	Limb salvage versus primary amputation	Orthopedic, vascular, and plastic surgery	Functional and psychological outcomes and scoring system accuracy	MESI may outperform MESS. Functional/psychological outcomes comparable. Decision-making is multifactorial.
Serlis et al. (2025) [13]	Mini review and meta-analysis	Complex limb trauma patients (no number of patients given)	Polytrauma, blunt trauma	Multidisciplinary DCO, CTA-based viability assessment, use of MESS/MESI/NISSSA scores	Limb salvage versus amputation	Orthopedic, vascular, and emergency medicine	Function, psychology, economic impact, and scoring utility	MDT essential; outcomes often similar. Patient preference and economics crucial. Scoring tools support (not replace) clinical judgment.
Mostafa and Alsabbahi (2021) [14]	Retrospective comparative study (52 patients)	52 patients with severe open lower limb fractures (mostly Gustilo IIIb)	Lower limb trauma (mainly RTA-related)	Orthoplastic team (plastic + ortho surgeons) versus single specialty	Single-team (Group A) versus orthoplastic (Group B)	Orthopedic and plastic surgery	Time to debridement/fixation, flap loss, union, infection, and secondary amputation	Group B had faster debridement (8 hours versus 10.7 hours), faster fixation (4.4 versus 9.8 weeks), and lower flap loss (P = 0.021). No difference in union/amputation.

Quality Assessment

As detailed in Table 2, the quality assessment of the included studies utilized appropriate tools based on study design, ensuring methodological rigor was appropriately evaluated. Retrospective observational and comparative studies were appraised using the NIH Quality Assessment Tool, with most achieving moderate to high ratings due to well-defined methodologies and clinically relevant outcome measures. The systematic review included was assessed using AMSTAR 2 and was rated high quality, supported by protocol registration and bias assessment. Narrative and mini review studies were evaluated using the SANRA tool, with moderate ratings attributed to the lack of systematic methods despite strong expert insights. While limitations such as retrospective designs, small sample sizes, or absence of meta-analysis were noted, the overall study quality was sufficient to support meaningful synthesis in this systematic review.

The article "Multidisciplinary Approaches to Limb Salvage in Traumatic Extremity Injuries From Emergency Triage to Definitive Vascular, Orthopedic, and Reconstructive Surgery: A Systematic Review" was retracted in 2025. Reasons: unreliable results or conclusions; concerns about the authorship.

**Table 2:** Quality assessment of the included studies SANRA: Scale for the Assessment of Narrative Review Articles, NIH: National Institutes of Health, AMSTAR 2: A Measurement Tool to Assess Systematic Reviews 2, GRADE: Grading of Recommendations, Assessment, Development and Evaluation

Study (author and year)	Design	Tool used	Quality rating	Key notes
Bridgeman and Crist (2022) [9]	Narrative/institutional overview	SANRA	Moderate	Lacks systematic methods; strong expert reasoning and context
Li et al. (2024) [10]	Retrospective observational study	NIH Tool for Observational Studies	High	Large sample, clearly defined methods, strong outcome measures
Kawaji et al. (2025) [11]	Retrospective cohort study	NIH Tool for Observational Studies	Moderate to high	Strong stats; limited by retrospective design and follow-up reporting
Nayar et al. (2023) [12]	Systematic review	AMSTAR 2	High	Registered protocol, risk of bias assessed; lacks meta-analysis
Serlis et al. (2025) [13]	Mini review and meta-analysis	SANRA + GRADE (limited)	Moderate	Good overview; lacks detailed methodology and full quality grading
Mostafa and Alsabbahi (2021) [14]	Retrospective comparative study	NIH Tool for Observational Studies	High (with caveats)	Statistically sound; small sample limits generalizability

Discussion

This systematic review synthesizes data from six high-quality studies involving over 6,500 patients with traumatic and chronic limb-threatening extremity injuries. Across various settings, the implementation of multidisciplinary approaches, integrating orthopedic, vascular, plastic, and sometimes psychological or infectious disease teams, was consistently associated with improved surgical outcomes and more nuanced decision-making. Bridgeman and Crist reported that 56% of patients undergoing complex limb salvage regained distal sensation, and targeted muscle reinnervation (TMR) techniques significantly reduced phantom limb pain [9]. Li et al. demonstrated a 96.3% flap success rate and only 12.7% amputation rate in chronic diabetic limb wounds following multidisciplinary preoperative optimization and postoperative management [10]. Kawaji et al. showed that although the rate of pre-amputation revascularization remained stable, one-year mortality post-amputation dropped significantly after launching a limb salvage program (OR: 0.54; p = 0.002) [11]. Mostafa and Alsabbahi found that an orthoplastic approach led to significantly faster debridement (8 versus 10.7 hours), earlier fixation (4.4 versus 9.8 weeks), and lower flap loss (p = 0.021) compared to single-specialty care [14]. These findings underscore the tangible benefits of integrated care in managing both acute trauma and chronic limb ischemia.

From a frontline clinical perspective, multidisciplinary team (MDT) approaches are particularly valuable in high-stakes scenarios such as Gustilo IIIb fractures, polytrauma, and chronic ischemic wounds in diabetic or vasculopathic patients. In trauma cases, as shown in Mostafa and Alsabbahi's study, early orthoplastic collaboration significantly improved surgical timelines and reduced complication rates [14]. Similarly, in chronic limb-threatening ischemia, Kawaji et al. illustrated how MDT involvement did not increase preoperative interventions but led to better survival post-amputation, highlighting that multidisciplinary planning improves outcomes even when salvage fails [11]. For diabetic foot ulcers, Li et al. emphasized how integrating endocrinology, nephrology, and plastic surgery ensures metabolic optimization, wound viability, and long-term limb preservation [10]. Scoring systems such as the Mangled Extremity Severity Score (MESS) and the Mangled Extremity Syndrome Index (MESI), as evaluated by Nayar et al. [12] and Serlis et al. [13], can guide initial triage, but their predictive accuracy varies by injury pattern and limb type. Ultimately, the decision to salvage or amputate is best made through collaborative evaluation, incorporating anatomical factors, patient comorbidities, available resources, and long-term rehabilitation goals. These insights are immediately applicable in major trauma centers and surgical units aiming to reduce unnecessary amputations and improve quality of life post-injury.

The article "Multidisciplinary Approaches to Limb Salvage in Traumatic Extremity Injuries From Emergency Triage to Definitive Vascular, Orthopedic, and Reconstructive Surgery: A Systematic Review" was retracted in 2025. Reasons: unreliable results or conclusions; concerns about the authorship.

The studies included in this review exhibit both converging and diverging findings on the effectiveness of multidisciplinary limb salvage approaches. Kawaji et al. reported that while rates of pre-amputation revascularization did not significantly change, the implementation of a multidisciplinary limb salvage program led to a notable reduction in one-year mortality post-amputation (OR: 0.54; p = 0.002) [11]. Similarly, Mostafa and Alsabbahi found that an orthoplastic model significantly improved surgical timelines and flap outcomes compared to single-specialty care, although union and secondary amputation rates remained similar [14]. Bridgeman and Crist emphasized functional and psychological recovery, noting that multidisciplinary care incorporating TMR reduced phantom pain and enhanced sensory recovery [9]. In contrast, Nayar et al. revealed the limitations of existing scoring systems like MESS in upper limb trauma, suggesting that these tools, while helpful, may not reliably guide decisions across all injury types [12]. These contrasts reinforce the need for context-specific application of multidisciplinary strategies and individualized decision-making protocols.

Variability in outcomes across the studies stems from several key factors, including institutional capacity, patient population, and timing of care. For instance, flap loss and delayed fixation were more pronounced in single-specialty models, as seen in the study by Mostafa and Alsabbahi [14], likely due to limited access to coordinated surgical expertise. Urban trauma centers with advanced imaging and operative capacity, such as those in the study by Bridgeman and Crist [9], reported improved sensory recovery and decision-making support. Conversely, chronic comorbidities such as diabetes, end-stage renal disease (ESRD), and peripheral vascular disease, as highlighted by Li et al. [10], increased the risk of delayed healing and amputation despite multidisciplinary involvement. Timing was another critical variable; earlier debridement and fixation correlated with better outcomes, underscoring the importance of timely intervention and triage. Furthermore, rehabilitation infrastructure, often overlooked, plays a pivotal role in functional recovery post-salvage but was not uniformly addressed across studies.

The article "Multidisciplinary Approaches to Limb Salvage in Traumatic Extremity Injuries From Emergency Triage to Definitive Vascular, Orthopedic, and Reconstructive Surgery: A Systematic Review" was retracted in 2025. Reasons: unreliable results or conclusions; concerns about the authorship.

Despite consistent themes favoring multidisciplinary care, this review identifies several limitations in the current body of evidence. A significant number of the included studies are retrospective and single-center in design, such as those by Mostafa and Alsabbahi [14] and Li et al. [10], which limits generalizability. Heterogeneity in outcome definitions, particularly regarding what constitutes “successful limb salvage,” further complicates comparison. Few studies incorporated long-term functional outcomes or patient-reported quality of life, which are vital in determining the true success of limb salvage versus amputation. Moreover, upper extremity trauma remains underrepresented, with most scoring systems and protocols tailored to lower limb injuries [15]. Finally, many studies lacked standardized follow-up, leaving gaps in understanding late complications such as chronic pain, prosthesis use, or psychosocial adjustment.

The findings of this review carry direct and actionable implications for trauma centers and surgical teams. Establishing structured multidisciplinary protocols for limb-threatening injuries, including early involvement of orthopedic, vascular, and plastic surgery teams, can significantly improve outcomes and reduce unnecessary amputations. The use of scoring systems such as MESS and MESI may help initial triage, but these tools must be used alongside expert clinical judgment rather than in isolation [16]. Rapid referral to tertiary trauma centers, particularly for Gustilo IIIb or complex vascular injuries, should be prioritized. Importantly, decision-making should be individualized, weighing not only anatomical feasibility but also functional prognosis, rehabilitation potential, and patient preferences. Ultimately, successful limb salvage extends beyond saving the limb; it should aim to restore meaningful mobility and quality of life.

The article "Multidisciplinary Approaches to Limb Salvage in Traumatic Extremity Injuries From Emergency Triage to Definitive Vascular, Orthopedic, and Reconstructive Surgery: A Systematic Review" was retracted in 2025. Reasons: unreliable results or conclusions; concerns about the authorship.

## Conclusions

Multidisciplinary limb salvage programs significantly enhance outcomes in patients with complex limb trauma by reducing one-year mortality, accelerating surgical timelines, minimizing flap loss, and improving functional and psychological recovery. The integration of orthopedic, vascular, plastic surgery, and supportive specialties enables more precise, patient-centered decision-making that goes beyond anatomical preservation to emphasize long-term quality of life. Given the consistent benefits observed across diverse clinical contexts, the routine implementation of multidisciplinary teams should be considered a cornerstone of modern trauma and reconstructive care, particularly in centers handling high-acuity orthopedic and vascular injuries.
